# Antihypertension Induced by Tanshinone IIA Isolated from the Roots of *Salvia miltiorrhiza*

**DOI:** 10.1093/ecam/nep056

**Published:** 2011-01-04

**Authors:** Paul Chan, I-Min Liu, Ying-Xiao Li, Wen-Jen Yu, Juei-Tang Cheng

**Affiliations:** ^1^Division of Cardiovascular Medicine, Taipei Medical University-Wan Fang Hospital, Taipei City 11601, Taiwan; ^2^Department of Pharmacy, Tajen University, Yen-Pou, Ping Tung Shien 90701, Taiwan; ^3^Department of Hematology, Guangzhou First Municipal People's Hospital, Guangzhou City, China; ^4^Department of Biotechnology, Hung Kuang University, Sha Lu, Taichung Shien 43301, Taiwan; ^5^Department of Pharmacology, College of Medicine, National Cheng Kung University, Tainan City 70101, Taiwan

## Abstract

Tanshinone IIA is one of the active principles in danshen (*Salvia miltiorrhiza* Bge) widely used in treatment of cardiovascular disorders. We investigated the effect of danshen or tanshinone IIA on blood pressure and its possible mechanisms. An i.p. injection of danshen at 10 mg kg^−1^ significantly lowered systolic blood pressure (SBP) of spontaneously hypertensive rats (SHRs) but failed to modify the SBP in normotensive Wistar-Kyoto rats (WKY). Oral administration of tanshinone IIA also decreased SBP in SHR but not in WKY. Tanshinone IIA produced a concentration-dependent relaxation in isolated SHR aortic rings precontracted with phenylephrine (10 nmol l^−1^) or potassium chloride (KCl) (40 mmol l^−1^). The relaxing effect of tanshinone IIA on tonic contraction of phenylephrine in isolated aortic rings without endothelium remained produced. Glibenclamide at concentration sufficient to block adenosine triphosphatase (ATP)-sensitive potassium (K^+^) channel attenuated this tanshinone IIA-induced relaxation that was not influenced by other inhibitors. We further investigated the effect of tanshinone IIA on the changes of intracellular calcium concentration ([Ca^2+^]_*i*_) in cultured aortic smooth muscle (A7r5) cells using fura-2 as indicator. Tanshinone IIA decreased [Ca^2+^]_*i*_ elicited by phenylephrine (10 nmol l^−1^) or KCl (40 mmol l^−1^) in a concentration-dependent manner; glibenclamide, but not other inhibitors for K^+^ channel, abated this effect. Our results suggest that tanshinone IIA acts as an active principle of danshen showing vasodilation through ATP-sensitive K^+^ channel to lower [Ca^2+^]_*i*_.

## 1. Introduction

Danshen, the dry root and rhizome of *Salvia miltiorrhiza* Bge (Labiatae), is one of the popular herbs used in China and the neighboring countries. This herb is widely applied in traditional Chinese medicine for promotion of blood flow to overcome blood stasis and to resolve abscesses [1]. Many clinical studies showed that Danshen and its preparations are effective for the treatment of coronary artery diseases, angina pectoris, myocardial infarction, cerebrovascular diseases, various types of hepatitis and chronic renal failure [1–3]. In addition to the protection of cardiac muscle during angioplasty or heart transplantation, Danshen has also been recommended for treatments of menstrual disorder, insomnia as well as inflammation [4, 5].

Danshen and its medicinal products are widely used in Asian area for supporting cardiovascular function; evaluation of the active constituents in this herb is essential to ensure the efficiency of medication. Studies showed that this herb contains several pharmacologically active compounds, especially the diterpene diketones known as tanshinones [6]. This major active ingredient of Danshen is reported to work as a vasodilator, causing blood vessels to relax and increase blood circulation. Also, it has the ability to inhibit platelet aggregation, thereby reducing the risk of arteriosclerosis, stroke and heart attack [5]. Tanshinones seem to be the active ingredients of Danshen for cardioprotective effect.

Danshen has been mentioned to inhibit angiotensin-converting enzyme, an essential regulatory enzyme of rennin-angiotensin system, for lowering blood pressure [7]. In fact, the membrane potential is a major determinant of vascular tone; changes in potassium (K^+^) channel activity is responsible for the reduction of intracellular calcium ion concentrations ([Ca^2+^]_*i*_) to produce vasodilatation [8]. However, the effect of tanshinone on vascular tone involved in the changes of K^+^ conductance to regulate Ca^2+^ mobilization is still not established. Thus, the main aim of this study is to evaluate the effect of tanshinone IIA, one of the tanshinones, on blood pressure in rats with spontaneous hypertension and to characterize the effect of tanshinone IIA on vascular tone, using specific blockers of K^+^ channel to investigate the role of this channel in spontaneously hypertensive rat (SHR)-isolated aortic rings strips and cultured A7r5 vascular smooth muscle cells.

## 2. Methods

### 2.1. Materials

Danshen (voucher 0425) and tanshinone IIA with the purity of 98% was gifted from Prof. De-Yu Xu (Department of Pharmacology, College of Medicine, Nanjin University, Nanjin City, China). Acetylcholine, l-phenylephrine, potassium chloride, glibenclamide, apamin, charybdotoxin, barium chloride and 4-aminopyridine were obtained from Sigma-Aldrich, Inc. (St. Louis, MO, USA). Dulbecco's modified Eagle's medium (DMEM) was purchased from GIBCO BRL (Gaithersburg, MD). Fura-2 acetoxymethyl ester (fura-2) was from Molecular Probes Inc. (Eugene, OR, USA). All other reagents were obtained from standard sources.

### 2.2. Experimental Animals

We obtained 10-week-old male rats with SHR and age-matched male Wistar-Kyoto rats (WKY) from National Animal Center (Taipei, Taiwan) to keep in our animal center. Also, the male Wistar rats at same age from our animal center were employed. They were maintained in a temperature-controlled room (25°C ± 1) under a cycle of 12 h of light (beginning at 6:00 A.M.) and 12 h of darkness. All rats were given water and fed standard chow (Purina Mills, LLC, St Louis, MO, USA) *ad libitum*. All animal-handling procedures were performed according to the Guide for the Care and Use of Laboratory Animals of the National Institutes of Health as well as the guidelines of the Animal Welfare Act.

### 2.3. Measurement of Blood Pressure in Conscious Rats

The powder of danshen and compound of tanshinone IIA were dissolved in alcoholic solution (90%) and prepared with distilled water containing 0.9% sodium chloride immediately before use. Danshen solution at the indicated dose was given by an intraperitoneal (i.p.) injection into rats. Another group of rats were treated by an oral administration of tanshinone IIA solution at the desired dose. Control rats received similar administration of vehicle at same volume as that used in the treated rats.

Systolic blood pressure (SBP) in conscious rats was determined using a noninvasive tail-cuff monitor (MK2000; Muromachi Kikai Co. Ltd, Tokyo, Japan). Values are presented as the mean of three measurements.

### 2.4. Preparation of Isolated Aortic Rings

The application of aortic ring isolated from SHR was employed in the present study. Each rat was sacrificed by means of decapitation under anesthesia with pentobarbital (50 mg kg^−1^). As described in our previous study [9], we rapidly removed the thoracic aortae and placed them in oxygenated Krebs buffer (95% O_2_, 5% CO_2_). After the fat and connective tissue were gently dissected, the aortae were cut into ring segments approximately 3-mm long. The rings were then mounted in 37°C organ baths filled with 10 mL of oxygenated Krebs buffer (95% O_2_, 5% CO_2_) containing 135 mmol l^−1^ NaCl, 5 mmol l^−1^ KCl, 2.5 mmol l^−1^ CaCl_2_, 1.3 mmol l^−1^ MgSO_4_, 1.2 mmol l^−1^ KH_2_PO_4_, 20 mmol l^−1^ NaHCO_3_ and 10 mmol l^−1^ d-glucose (pH 7.4).

Each preparation was connected to strain gauges (FT03; Grass Instrument Co., Quincy, MA, USA). Isometric tension was recorded by using chart software (MLS023, Powerlab; AD Instruments Pty Ltd, Bella Vista, New South Wales, Australia). The rings were mounted and allowed to stabilize for 2 h. The preparation was then gradually stretched to achieve an optimal resting tension of 1 g.

### 2.5. Removal of Endothelium

To preclude the possible role of endothelium in the vasodilatation of tanshinone IIA, the tests were conducted in endothelium-denuded preparations. The endothelium was removed by gently rubbing against the teeth of a pair of forceps. Success of the removal of endothelium was characterized using the failure of 10 *μ*mol l^−1^ acetylcholine to relax the rings precontracted with 10 nmol l^−1^ phenylephrine.

### 2.6. Vasodilatation Induced by Tanshinone IIA

After stabilization of resting tension, phenylephrine (10 nmol l^−1^) or potassium chloride (KCl) (40 mmol l^−1^) in distilled water was added into bathing buffer to induce a rapid increase in vascular tone followed by stable vasoconstriction (tonic contraction). The treatment group was given tanshinone IIA (0.1–10 *μ*mol l^−1^) to observe the decrease in tonic contraction (vasodilatation). Relaxation was expressed as the percentage decrease of maximal tonic contraction. Concentration-relaxation curves were generated in cumulative fashion.

### 2.7. Effect of K^+^ Channel Blockers on the Vasodilatation of Tanshinone IIA

After the resting tension became stabilized, phenylephrine (10 nmol l^−1^) or KCl (40 mmol l^−1^) was administered into bathing buffer to induce an increase of vascular tone followed by the stable vasoconstriction (tonic contraction). Then, testing groups were treated with tanshinone IIA to produce a lowering of tonic contraction that was indicated as vasodilatation in the present study. The K^+^ channel blockers, including glibenclamide, apamin, charybdotoxin, barium chloride and 4-aminopyridine, dissolved in distilled water, were administered at the effective concentration for 30 min before tanshinone IIA was added and the vasodilatation of tanshinone IIA was compared with samples treated same volume of vehicle used to dissolve the testing blockers [9, 10]. The relaxation was calculated from the decrease of tonic vasoconstriction induced by phenylephrine or KCl and expressed as the percentage of maximal contraction. Concentration-relaxation curves were generated in a cumulative fashion.

### 2.8. Measurement of [Ca^2+^]_*i*_ Concentration in A7r5 Cells with Fura-2

The A7r5 line of rat aortic smooth muscle cells obtained from the Food Industry Institute (Hsin-Chu, Taiwan) were incubated in DMEM containing 10% (V V^−1^) fetal bovine serum with fura-2 (5 *μ*mol l^−1^) in the dark at room temperature for 30 min. Then, the cells were gently washed twice with Ca^2+^-free physiologic salt solution after they were centrifuged at 3000 rpm for 7 min and kept in the same solution containing Ca^2+^. The physiologic salt solution contained 140 mmol l^−1^ NaCl, 5.9 mmol l^−1^ KCl, 1.2 mmol l^−1^ NaH_2_PO_4_, 5 mmol l^−1^ NaHCO_3_, 1.4 mmol l^−1^ MgCl_2_, 1.8 mmol l^−1^ CaCl_2_ and 11.5 mmol l^−1^ glucose. The cells were maintained on ice until the [Ca^2+^]_*i*_ was measured.

The [Ca^2+^]_*i*_ was measured by using an emission wavelength of 520 nm and alternating excitatory wavelengths of 340 and 380 nm (F-2000 spectrophotometer; Hitachi, Tokyo, Japan). Using external calibration, we then calculated [Ca^2+^]_*i*_ according to the equation [Ca^2+^]_*i*_ = [(*R* − *R*_min_)/(*R*_max_ − *R*)×(*S*_f2_/*S*_b2_)×*K*_d_], where *R* is the fluorescence intensity of the Ca^2+^-sensitive dye fura-2 at excitation wavelengths of 340 and 380 nm, *R*_min_ is the minimum fluorescence ratio of about 0.768 and *R*_max_ is the maximum fluorescence ratio of about 35.1. The coefficient *S*_f2_ indicates the free dye measured at wavelength of 380 nm and *S*_b2_ indicates Ca^2+^-bound dye at 380 nm. According to experimental data, *S*_f2_/*S*_b2_ for fura-2 is about 15.3. *K*_d_ is the effective dissociation constant of fura-2, which was about 135 nmol l^−1^.

The change of [Ca^2+^]_*i*_ in response to phenylephrine or KCl was evaluated by using normal physiologic salt solution containing Ca^2+^. Pretreatment of tanshinone IIA was carried out to identify its antagonism of Ca^2+^. We administered the K^+^ channel blockers, then added tanshinone IIA to determine this inhibition of [Ca^2+^]_*i*_ by tanshinone IIA that involved the opening of K^+^ channels.

### 2.9. Statistical Analysis

Data were expressed as the mean ± SD for the number (*n*) of animals in each group as indicated in the tables and figures. Statistical differences among groups were determined by using two-way repeated-measure ANOVA. Dunnett range post-hoc comparisons were used to determine the source of significant differences where appropriate *P*  value < .05 was considered statistically significant.

## 3. Results

### 3.1. Danshen-Induced Modulation of SBP in Rats

A dose-dependent decrease of SBP in SHR received an i.p. injection of danshen was shown in Figure 1; the maximal effect (20.1 ± 3.1%) was achieved by 60-min treatment with danshen at 10 mg kg^−1^. The effect of danshen on the reduction of SBP was maintained for 150 min (Figure 1). No change of SBP was observed in WKY receiving the similar administration of danshen at 10 mg kg^−1^ for 60 min (Figure 1).

### 3.2. Tanshinone IIA-Induced Modulation of SBP in SHR

After treatment with tanshinone IIA, SBP was noticeably reduced in SHR; a 60-min treatment with tanshinone IIA at the oral dosage of 60 mg kg^−1^ significantly lowered SBP in SHR (Figure 2) However, administering WKY with tanshinone IIA (60 mg kg^−1^) for 60 min failed to modify the SBP (Figure 2).

### 3.3. Tanshinone IIA-Induced Changes on Vascular Tone

The SHR aortic ring strips strongly contracted after an initial application of phenylephrine (10 nmol l^−1^) or KCl (40 mmol l^−1^) (Figure 3). Although tanshinone IIA did not influence resting vascular tone, it dilated both phenylephrine- and KCl-induced contractions in a concentration-dependent manner. At the maximal concentration, tanshinone IIA (10 *μ*mol l^−1^) significantly attenuated the tonic contraction of SHR aortic rings induced by phenylephrine (10 nmol l^−1^) to 24.9 ± 5.2% of the maximal contraction (Figure 3). Also, the effect of tanshinone IIA (10 *μ*mol l^−1^) on KCl (40 mmol l^−1^)-induced tonic vasoconstriction approached 28.3 ± 5.4% of the maximal contraction (Figure 3).

### 3.4. Role of Endothelium in Tanshinone IIA-Induced Relaxation

No difference (*P* > .05) can be observed regarding the relaxing effect of tanshinone IIA (10 *μ*mol l^−1^) on phenylephrine (10 nmol l^−1^)-induced tonic vasoconstriction between SHR aortic rings with or without functional endothelium (Figure 4).

### 3.5. Role of K^+^ Channels in Tanshinone IIA-Induced Vasodilatation

In the presence of glibenclamide (1–100 *μ*mol l^−1^), the blockers specific to ATP-sensitive K^+^ (K_ATP_) channel, the relaxing effect of tanshinone IIA on tonic contraction in phenylephrine (10 nmol l^−1^)-precontracted SHR aortic rings was significantly reduced in a concentration-dependent manner (Table 1). The vasodilatation due to tanshinone IIA in KCl (40 mmol l^−1^)-pretreated SHR aortic rings was also attenuated under glibenclamide treatment in a similar way (Table 1).

However, in the presence of a blocker specific to the Ca^2+^-sensitive small conductance K^+^ (SK_Ca_) channel (0.1 *μ*mol l^−1^ apamin), the relaxing effect of tanshinone IIA on tonic contraction of phenylephrine (10 nmol l^−1^) remained at 25.1 ± 4.6% of the maximal contraction. Also, charybdotoxin (0.1 *μ*mol l^−1^), the large-conductance Ca^2+^-activated K^+^ channel (LK_Ca_ channel) blocker, failed to modify the relaxation of tanshinone IIA, with a result of 23.7 ± 5.2% of phenylephrine (10 nmol l^−1^)-induced tonic contraction. Moreover, inhibition of inward rectifier K^+^ channel (K_IR_ channel) with barium chloride (10 *μ*mol l^−1^) or blockade of voltage-dependent K^+^ channel (K_V_ channel) with 4-aminopyridine (1 mmol l^−1^), the relaxing effect of tanshinone IIA on tonic contraction of phenylephrine (10 nmol l^−1^) was still 26.4 ± 4.2% or 24.4 ± 6.5%, respectively (Table 1).

Similarly, the vasodilation due to tanshinone IIA in KCl (40 mmol l^−1^)-pretreated SHR aortic rings was not reserved under apamin treatment (Table 1). Also, blockade of LK_Ca_, K_IR_ or K_V_ channel by other specific inhibitors failed to modify the vasodilatation of tanshinone IIA on KCl (40 mmol l^−1^)-induced tonic contraction (Table 1).

### 3.6. Role of K^+^ Channels in the Inhibitory Effect of Tanshinone IIA on Intracellular Ca^2+^ Concentrations in A7r5 Cells

In Ca^2+^-containing medium, phenylephrine (10 nmol l^−1^) increased [Ca^2+^]_*i*_ in A7r5 cells from 214.7 ± 34.2 to 440.2 ± 29.3 nmol l^−1^ (Figure 5). Tanshinone IIA attenuated this increase of [Ca^2+^]_*i*_ induced by phenylephrine (10 nmol l^−1^) in a concentration-dependent manner; the maximal inhibitory activity of tanshinone IIA was observed at 10 *μ*mol l^−1^ (Figure 5). However, glibenclamide (1–100 *μ*mol l^−1^) reversed the inhibitory effect of tanshinone IIA (10 *μ*mol l^−1^) on [Ca^2+^]_*i*_ induced by phenylephrine (10 nmol l^−1^) (Table 2).

Also, KCl (40 mmol l^−1^) increased [Ca^2+^]_*i*_ in A7r5 cells to 428.6 ± 27.4 nmol l^−1^ in Ca^2+^-containing medium (Figure 5). Tanshinone IIA similarly inhibited the elevation of [Ca^2+^]_*i*_ induced by KCl (40 mmol l^−1^) in a concentration-dependent manner (0.1–10 *μ*mol l^−1^) parallel to its effects against the action of phenylephrine (10 nmol l^−1^) (Figure 5), though glibenclamide markedly attenuated this effect (Table 2).

However, neither apamin (0.1 *μ*mol l^−1^) nor charybdotoxin (0.1 *μ*mol l^−1^) modify the inhibition of tanshinone IIA (10 *μ*mol l^−1^)-induced changes in [Ca^2+^]_*i*_ in A7r5 cells; the rise of [Ca^2+^]_*i*_ in A7r5 cells by phenylephrine (10 nmol l^−1^) or KCl (40 mmol l^−1^) was not changed significantly (Table 2). Also, barium chloride (10 *μ*mol l^−1^) or 4-aminopyridine (1 mmol l^−1^) did not influence the inhibitory effect of tanshinone IIA on [Ca^2+^]_*i*_ in phenylephrine (10 nmol l^−1^)- or KCl (40 mmol l^−1^)-treated A7r5 cells (Table 2).

## 4. Discussion

Clinically, the application of danshen is clearly studied and intravenous injection danshen containing 40 mg of tanshinone IIA twice a day for 28 days is effective to improve the neurological functions in patients suffered with strokes [5]. Also, oral administration of tanshinone IIA at 1 g daily doses is helpful to cure the stroke symptoms [5]. Danshen and the contained activate compounds, tanshinone IIA, may potentially provide advantage on the control of cardiovascular diseases in clinic. Tanshinone IIA has been introduced as the most abundant and representative principle of tanshinone derivatives [11], while tanshinone IIA is rapidly cleared by hepatic metabolism and cryptotanshinone is converted into tanshinone IIA as a precursor in the liver [12]. In the present study, we found that danshen and tanshinone IIA markedly decreased blood pressure in hypertensive rats, but the benefit effects on the regulation of blood pressure were not exited in the normotensive rats. Thus, we used tanshinone IIA to evaluate the vasodilative activity in isolated aorta to support the blood pressure lowering the efficacy of danshen in hypertensive rats, mainly mediated by the action of tanshinone IIA. Tanshinone IIA as the active ingredient in danshen for cardiovascular diseases was further supported by finding that phenylephrine- or KCl-induced tonic contraction in aortic ring prepared from hypertensive rats was alleviated by tanshinone IIA. Further research seems essential to understand the action mechanisms of tanshinone IIA for aortic relaxation.

Role of the endothelium in controlling vascular contractility is well established and dysfunction of arterial tone is believed to be due to abnormal endothelial function and/or reduced nitric oxide (NO) in vascular disease [13, 14]. It has been documented that danshen acts partially through endothelial nitric oxide synthase-signaling mechanisms to induce vasodilation and reduce blood pressure in hypertensive hamsters [15]. However, vasodilatation of tanshinone IIA remained produced in the absence of endothelium; the endothelium-dependent NO-mediated vasodilation seems unlikely to be involved in the antihypertensive action of tanshinone IIA. In general, an increase of [Ca^2+^]_*i*_ is considered as the major event of contraction in smooth muscle cells; blockade of Ca^2+^ channels is the most common factor in antihypertensive or vasodilative effects [16]. We observed that tanshinone IIA reduced phenylephrine- or KCl-induced elevation of [Ca^2+^]_*i*_ in cultured aortic smooth muscle cells, indicating that reduction in [Ca^2+^]_*i*_ might be related to the vasodilative effect of tanshinone IIA.

It is well known that membrane potential is a major determinant of vascular tone and K^+^ channels play an important role in the regulation of membrane potential in vascular smooth muscle [8]. Changes in the activity of K^+^ channels in vascular smooth muscle cell to elicit hyperpolarization and thereby a decline in [Ca^2+^]_*i*_ may result in vasodilatation [8, 16]. Therefore, we investigated the role of K^+^ channel in tanshinone IIA-induced vasorelaxation.

The family of K^+^ channels is at least five well-characterized members; the ATP-sensitive K channel is likely to be a temporarily activated K^+^ channel that may influence the [Ca^2+^]_*i*_ related to the regulation of vascular tone in vascular smooth muscle [8, 17]. It has been documented that KCl at the concentration <50 mmol l^−1^ did not depolarize the membrane via opening of ATP-sensitive K^+^ channels [18]. Actually, we used KCl at 40 mmol l^−1^ to depolarize the membrane of A7r5 cells and it is tanshinone IIA sensitive. We then investigated the role of K^+^ channels in the action of tanshinone IIA using pharmacologic blockers. In the presence of effective concentration of glibenclamide, the well-known ATP-sensitive channel blocker [18], the ability of tanshinone IIA to relax tonic contraction of isolated SHR aortic rings was ablated. Glibenclamide also blunted the decrease of [Ca^2+^]_*i*_ due to tanshinone IIA in phenylephrine- or KCl-pretreated A7r5 cells. However, apamin (SK_Ca_ channel blocker), charybdotoxin (LK_Ca_ channel blocker), barium chloride (K_IR_ channel blocker) and 4-aminopyridine (K_V_ channel blocker) were unable to interfere the ability of tanshinone IIA to relax tonic contraction of aortic rings isolated from SHR [13, 19, 20]; these inhibitors also failed to modify the inhibitory effect of tanshinone IIA on the elevation of [Ca^2+^]_*i*_ induced by phenylephrine or KCl. Thus, the effect of tanshinone IIA on vasodilatation is not expected to be related to SK_Ca_, LK_Ca_, K_IR_ or K_V_ channels; selective opening of ATP-sensitive K^+^ channels can thus be considered for the action of tanshinone IIA regarding the reduction of [Ca^2+^]_*i*_ to produce vasodilatation. Thus, it could be speculated that tanshinone IIA poses the ability to open ATP-sensitive K^+^ channels, which in turn leads to diffusion of K^+^ ions out of the vascular smooth muscle cells, then causes membrane hyperpolarization to close voltage-gated Ca^2+^ channels, thus resulting in decreased [Ca^2+^]_*i*_, and ultimately leads to vasodilatation (Figure 6).

In fact, glibenclamide attenuated but did not abolish the action of tanshinone IIA. Activation of ATP-sensitive K^+^ channels appeared to be involved, cannot account entirely for the vasodilative action of tanshinones. The increase in [Ca^2+^]_*i*_ reflects both the influx of Ca^2+^ and the release of Ca^2+^ from subcellular stores [21]. It has been demonstrated that the relaxation effects of danshen and its lipid-soluble components (tanshinone I, tanshinone II(A), cryptotanshinone, dihydroisotanshinone I) and the water-soluble compounds (danshensu and salvianolic acid B) on the isolated rat femoral artery were produced by inhibition of Ca^2+^ influx while a small component was mediated by the opening of K^+^ channels [22]. Also, sodium pumping or a pH-sensitive twin-pore domain K^+^ channel contributes in the membrane hyperpolarization [23, 24]. Therefore, other mechanisms responsible for tanshinone-induced lowering of [Ca^2+^]_*i*_ in addition to the opening of ATP-sensitive K^+^ channel should be considered.

Nonetheless, it has been indicated that distribution and/or sensitivity of ATP-sensitive K^+^ channel increased in the hypertensive state to result in an augmented relaxation to ATP-sensitive K^+^ channel opener which may be one of the compensatory mechanisms to maintain vasorelaxation in disordered state where endothelial function is impaired [25]. Also, vasorelaxation in response to ATP-sensitive K^+^ channel opener was augmented in arteries from hypertensive rats comparing to those from normotensive rats [7]. In the present study, tanshinone IIA did not influence the resting vascular tone but reduced the vasoconstriction only. Also, the chemical structure of tanshinone IIA is different with catecholamine; mediation of sympathetic nervous parameters in this action of tanshinone IIA could be ruled out. This is helpful to explain why tanshinone IIA lowered BP in SHR but not in WKY.

It has been indicated that tanshinone derivatives including cryptotanshinone and 15,16-dihydrotanshinone I are the important constituents for the use of danshen in inflammatory conditions [26]. Inhibition of osteoclast differentiation by available tanshinone such as diterpenoids, tanshinone I, tanshinone IIA, cryptotanshinone and dihydrotanshinone has also been demonstrated [27]. However, the evidence of active ingredients for the efficacy of danshen in cardiovascular disease has some limitations. Our results provided new insight for the application of tanshinone IIA in opening ATP-sensitive K^+^ channels, an effect which might be useful for the understanding of action and mechanisms of danshen in producing aortic relaxation. Indeed, ATP-sensitive K^+^ channel openers are vasodilators used in clinic [28]. The herbal principle, such as tetramethylpyrazine, an active ingredient found in the herb *Ligusticum chuanxiong* Hort. (Umbelliferae), is similar to tanshinone IIA acting as the ATP-sensitive K^+^ channel opener [9, 10]. Thus, herbal products responsible for the opening of ATP-sensitive K^+^ channels might eventually be useful in the handling of hypertension and/or cardiovascular disorders.

In conclusion, the opening of ATP-sensitive K^+^ channels can be considered as one of the mechanisms for tanshinone IIA that reduced [Ca^2+^]_*i*_ to induce vasodilatation.

## Figures and Tables

**Figure 1:** Changes of SBP in WKY or SHR receiving an i.p. of danshen or vehicle at various times. Data were expressed as the mean ± SD for seven rats in each group. **P < .01 versus data from vehicle-treated WKY. ^#^ *P* < .05 and ^##^ *P* < .01 versus vehicle-treated SHR, respectively.

**Figure 2:** Changes of SBP in WKY or SHR receiving an oral administration of tanshinone IIA or vehicle for 60 min. Data were expressed as the mean ± SD for seven rats in each group. **P < .01 versus data from vehicle-treated WKY. ^#^ *P* < .05 and ^##^ *P* < .01 versus vehicle-treated SHR, respectively.

**Figure 3:** Concentration-dependent relaxing action of tanshinone IIA in the isolated SHR aortic rings contracted with phenylephrine (10 nmol l^−1^) or KCl (40 mmol l^−1^). The preparation of isolated aortic rings from male SHR was described in Section 2. Data (mean ± SD) indicate the percentage dilations of the maximal contractions in eight experiments. *P < .05 and **P < .01 versus vehicle-treated group in each group.

**Figure 4:** Comparison of the dilative effect of tanshinone IIA on vasoconstriction induced by phenylephrine (10 nmol l^−1^) in the presence of endothelium (closed circle) or not (open circle). +, presence; –, absence. The preparation of isolated aortic rings from male SHR was described in Section 2. Data (mean ± SD) were obtained from eight experiments.

**Figure 5:** Effect of tanshinone IIA on the phenylephrine (10 nmol l^−1^) or KCl (40 mmol l^−1^)-induced increase of [Ca^2+^]_*i*_ in A7r5 line of rat aortic smooth muscle cells. Changes of [Ca^2+^]_*i*_ in A7r5 cells were measured by fura-2 as described in Section 2. The [Ca^2+^]_*i*_ obtained from A7r5 cells without treatment was 212.6 ± 32.4 nmol l^−1^. The data (mean ± SD) were obtained from six experiments.

**Figure 6:** Schematic mechanisms for the induction of vasodilatation by tanshinone IIA.

**Table 1:** Inhibitory effect of K^+^ channel blockers on the vasodilatation of tanshinone IIA in isolated SHR aortic rings contracted with phenylephrine or KCL^a^.

	Contraction force (%)			
	Phenylephrine (10 nmol l^−1^)		KCl (40 mmol l^−1^)	
	Vehicle	Tanshinone IIA (10 *μ*mol l^−1^)	Vehicle	Tanshinone IIA (10 *μ*mol l^−1^)
Basal	100^##^	24.9 ± 5.1**	100^##^	28.3 ± 4.8**
Glibenclamide (*μ*mol l^−1^)				
1	99.2 ± 4.9^*##*^	59.3 ± 7.1**	98.6 ± 5.8^*##*^	53.5 ± 4.9**
10	98.8 ± 6.1^*##*^	73.3 ± 5.9^∗,*#*^	98.2 ± 4.9^*##*^	78.6 ± 6.4^∗,*#*^
100	98.6 ± 5.6^*##*^	87.4 ± 6.7^*##*^	97.9 ± 6.3^*##*^	90.3 ± 5.6^*##*^
Apamin (0.1 *μ*mol l^−1^)	99.2 ± 3.7^*##*^	27.6 ± 4.7**	98.4 ± 4.7^*##*^	29.5 ± 5.7**
Charybdotoxin (0.1 *μ*mol l^−1^)	98.7 ± 4.1^*##*^	26.4 ± 5.1**	98.6 ± 5.3^*##*^	31.2 ± 4.9**
Barium chloride (10 *μ*mol l^−1^)	99.1 ± 5.6^*##*^	28.2 ± 3.9**	97.8 ± 4.6^*##*^	30.5 ± 5.1**
4-Aminopyridine (1 mmol l^−1^)	98.6 ± 3.9^*##*^	27.9 ± 4.2**	98.5 ± 6.9^*##*^	32.5 ± 6.1**

^a^The preparation of isolated aortic rings from male SHR was described in Section 2. Data (mean ± SD) indicate the percentage dilations of the maximal contractions in eight experiments. Data from phenylephrine (10 nmol l^−1^)- or KCl (40 mmol l^−1^)-treated sample without K^+^ channel blockers treatment was served as basal level in each group. *P < .05 and *P < .01 versus basal level obtained from samples treated with the same volume of vehicle to dissolve testing K^+^ channel blockers in each group. ^#^ *P* < .05 and ^##^ *P* < .01 versus value from sample received tanshinone IIA treatment in the absence of K^+^ channel blockers in each group.

**Table 2:** Effect of K^+^ channel blockers on the inhibition of tanshinone IIA-induced changes in [Ca^2+^]_*i*_ in A7r5 cells^a^.

	[Ca^2+^]_*i*_ (nmol l^−1^)			
	Phenylephrine (10 nmol l^−1^)		KCl (40 mmol l^−1^)	
	Vehicle	Tanshinone IIA (10 *μ*mol l^−1^)	Vehicle	Tanshinone IIA (10 *μ*mol l^−1^)
Basal	440.2 ± 29.3^*##*^	256.4 ± 32.5**	423.7 ± 32.4^*##*^	246.5 ± 27.6**
Glibenclamide (*μ*mol l^−1^)				
1	451.3 ± 35.7^*##*^	292.1 ± 27.6**	429.7 ± 37.2^*##*^	283.5 ± 29.8**
10	458.7 ± 30.2^*##*^	371.6 ± 23.7^∗,*##*^	432.6 ± 33.2^*##*^	386.2 ± 31.5^∗,*##*^
100	462.6 ± 32.3^*##*^	405.3 ± 31.4^*##*^	440.5 ± 34.6^*##*^	418.6 ± 28.6^*##*^
Apamin (0.1 *μ*mol l^−1^)	459.5 ± 39.2^*##*^	264.8 ± 28.4**	439.8 ± 29.7^*##*^	254.3 ± 27.2**
Charybdotoxin (0.1 *μ*mol l^−1^)	460.3 ± 34.2^*##*^	257.2 ± 26.7**	441.2 ± 31.4^*##*^	252.9 ± 30.6**
Barium chloride (10 *μ*mol l^−1^)	456.7 ± 33.9^*##*^	270.7 ± 32.4**	436.5 ± 28.6^*##*^	261.7 ± 25.9**
4-Aminopyridine (1 mmol l^−1^)	462.5 ± 30.1^*##*^	262.3 ± 34.1**	443.8 ± 32.5^*##*^	258.3 ± 28.6**

^a^Data (mean ± SD) were obtained from six experiments. The [Ca^2+^]_*i*_ obtained from A7r5 cells without any treatment was 214.7 ± 34.2 nmol l^−1^. Data from phenylephrine (10 nmol l^−1^)- or KCl (40 mmol l^−1^)-treated cells without K^+^ channel blockers treatment were served as basal level in each group. *P < .05 and **P < .01 versus basal level obtained from cells treated with the same volume of vehicle to dissolve testing K^+^ channel blockers in each group. ^#^ *P* < .05 and ^##^ *P* < .01 versus value from cells received tanshinone IIA treatment in the absence of K^+^ channel blockers in each group.
